# Supervised Learning Algorithm for Multilayer Spiking Neural Networks with Long-Term Memory Spike Response Model

**DOI:** 10.1155/2021/8592824

**Published:** 2021-11-24

**Authors:** Xianghong Lin, Mengwei Zhang, Xiangwen Wang

**Affiliations:** College of Computer Science and Engineering, Northwest Normal University, Lanzhou 730070, China

## Abstract

As a new brain-inspired computational model of artificial neural networks, spiking neural networks transmit and process information via precisely timed spike trains. Constructing efficient learning methods is a significant research field in spiking neural networks. In this paper, we present a supervised learning algorithm for multilayer feedforward spiking neural networks; all neurons can fire multiple spikes in all layers. The feedforward network consists of spiking neurons governed by biologically plausible long-term memory spike response model, in which the effect of earlier spikes on the refractoriness is not neglected to incorporate adaptation effects. The gradient descent method is employed to derive synaptic weight updating rule for learning spike trains. The proposed algorithm is tested and verified on spatiotemporal pattern learning problems, including a set of spike train learning tasks and nonlinear pattern classification problems on four UCI datasets. Simulation results indicate that the proposed algorithm can improve learning accuracy in comparison with other supervised learning algorithms.

## 1. Introduction

Research in neuroscience has shown that the precise timing of spikes (temporal encoding) is used to represent, transmit, and process information in the biological nervous system. The temporal encoding strategy can integrate many aspects of neural information, such as time, space, frequency, phase, etc. [1, 2]. The spiking neuron model is the basic computational units of spiking neural networks (SNNs), where precisely timed spikes are used to transmit the neural information [3, 4]. SNNs provide much greater computing capacity than the traditional artificial neural networks (ANNs) that employ the spike firing rate to encode neural information (rate encoding) [5]. SNN is a novel brain-inspired computational model and can efficiently deal with the spatiotemporal spike pattern learning problems [6, 7].

SNN computing and learning model plays an important role for brain-inspired artificial intelligence. In recent years, many supervised learning algorithms have been presented for different SNN architecture using various mechanisms [8]. Supervised learning of SNNs has been set up to find a suitable set of parameters (e.g., synaptic weight and synaptic delay) so that the network output spike trains that are highly similar to the given desired ones. In fact, neural information of SNNs is expressed in the form of discrete spike trains, and the neuronal internal state variables and network error function no longer meet the continuous differentiability. The traditional learning algorithm of ANNs, such as the error backpropagation algorithm [9], cannot be directly adopted for SNNs. Therefore, the formulation of efficient supervised learning algorithms for SNNs is difficult and remains an important problem in the research area.

According to the error backpropagation idea of traditional ANNs, researchers have proposed many gradient descent learning algorithms for multilayer feedforward SNNs. These algorithms use the gradient calculation and error backpropagation mechanism to design the synaptic weight updating rule to minimize the network error. In contrast to the neuron models expressed in the form of differential equations, the spike response model (SRM) is represented by the analytical expression with the kernel functions [10]. For this reason, SRM is usually adopted to construct SNNs and deduce the gradient descent learning rules. Bohte et al. [11] firstly reported a backpropagation supervised learning method, named SpikeProp. Through the learning of synaptic weights of SNNs, it shows that SpikeProp algorithm has the ability to solve nonlinear pattern classification problems, such as XOR problem. The SpikeProp algorithm has been improved and extended from different aspects [12, 13]. However, the SpikeProp algorithm and its simple extensions use single spike to encode information; that is, all neurons can only fire one spike in the process of network simulation. This limitation makes SpikeProp algorithm unable to solve complex problems effectively. More importantly, Xu et al. [14] proposed multi-SpikeProp algorithm; the gradient descent learning rules of synaptic weights in output and hidden layers are deduced by using chain rules. The algorithm has no restriction on the spike emissions of neurons in the network. However, the short-term memory SRM (abbreviated as SRM_0_) is used in the above algorithms, the membrane potential of SRM_0_ model depends only on the contribution of the most recent spike to refractoriness.

The leaky integrate-and-fire model is regarded as one of the most famous spiking neuron computational models. The SRM neuron model can be seen as a generalization form of the leaky integrate-and-fire model. It not only considers the spike trains transmitted by the presynaptic neurons, but also sums up all the spikes fired by itself. Therefore, the cumulative SRM model depends on all firing times of the neuron that contribute to refractoriness; it has a long-term memory feature [15]. The advantage of long-term memory SRM is that it can express the bursting and adaptation characteristics [16]. Booij and tat Nguyen [17] proposed a supervised learning algorithm for multilayer feedforward SNNs with long-term memory SRM. However, in this algorithm, neurons in the output layer are still limited to learn single spike. Spike trains encode significant neural information in the brain and the information cannot be simply represented by single spike. In order to simulate the activity of brain, it is necessary to study spike train supervised learning algorithm for multilayer feedforward SNNs. The design of spike train learning algorithm is more difficult than that of the single-spike learning for SNNs, but it has more powerful learning capability for solving the complex problems. Therefore, in this paper, combining with the long-term memory characteristic of SRM, we extend the algorithm proposed by Booij and tat Nguyen [17] and propose a supervised learning algorithm based on the error backpropagation of multiple spikes, which can achieve spike train learning for multilayer feedforward SNNs.

The rest of this paper is organized as follows.  Section 2 introduces the related works including the different supervised learning algorithms for SNNs.  Section 3 introduces the long-term memory SRM and the structure of feedforward SNNs used in this paper.  Section 4 deduces the supervised learning rules based on gradient descent, and the computational complexity of the proposed algorithm is also analyzed.  Section 5 demonstrates the performance of feedforward SNNs trained with the proposed learning algorithm through a series of spike train learning tasks and nonlinear pattern classification problems.  Section 6 concludes this paper.

## 2. Related Works

Supervised learning of ANNs is that neurons produce desired output for the given labelled data. In addition, researchers have considered the deep structure of the network [18, 19] and the multidirectional long short-term memory model [20]; the supervised learning is deeply investigated and applied to the engineering problems. In fact, experimental studies have shown that supervised learning exists in biological nervous systems, especially sensorimotor networks and sensory systems [21], but there is no clear conclusion on how biological neurons realize this process. Based on temporal encoding of SNNs, the learning methods have been introduced in recent years [22, 23]. According to the different ideas of supervised learning for multilayer feedforward SNNs, we divide the supervised learning algorithms into three categories.

### 2.1. Supervised Learning Algorithms Based on Gradient Descent Rule

Gradient descent method plays a prominent part in training networks with spiking neurons. The basic idea of gradient descent algorithms is to use the gradient value of the error between the desired and actual output spike trains as the reference for synaptic weight adjustment and ultimately reduce the network error. Although the gradient descent learning algorithms can be applied to multilayer feedforward SNN structure through error backpropagation mechanism, the state variables of neuron model must have analytical expressions, such as the leaky integrate-and-fire and SRM neuron models.

The SpikeProp [11] and its extended algorithms [14, 17, 24, 25] are typical gradient descent algorithms. In addition, Mostafa [26] derived a gradient descent training method of SNNs for processing spike patterns with realistic temporal dynamics. For the feedforward SNN with temporal coding scheme, the network input-output relation is piecewise linear after the variable transformation; the traditional ANN gradient descent technique is transferred to the SNN. By using the surrogate gradient approach, Zenke and Ganguli [27] proposed SuperSpike learning algorithm. A three-factor learning rule based on nonlinear voltage is capable of training multilayer feedforward networks with deterministic integrate-and-fire neurons, which can perform nonlinear computation on spatiotemporal spike patterns.

### 2.2. Supervised Learning Algorithms Based on Synaptic Plasticity Mechanism

Spike trains can not only cause continuous changes of synapses, but also meet the mechanism of spike timing-dependent plasticity (STDP) [28]. In a time window, when postsynaptic neuronal spike fires after presynaptic neuronal spike, it always causes long-term potentiation. On the contrary, it always causes long-term depression. STDP provides an experimental basis for the information strategy of spike-time coding and emphasizes the importance of asymmetry of spike-time correlations. Based on STDP mechanism, researchers have given a variety of supervised learning algorithms for SNNs. The basic idea of synaptic plasticity algorithms is to use the time correlation of presynaptic and postsynaptic spike trains for synaptic weight adjustment, which is a kind of supervised learning with biological interpretability.

Wade et al. [29] combined the Bienenstock–Cooper–Munro and STDP mechanisms and proposed a synaptic weight association training (SWAT) algorithm for multilayer feedforward SNNs. The stability of synaptic weight distribution is caused by modulated STDP plasticity window after a period of training. Ponulak and Kasiński [30] interpreted Widrow–Hoff rule as the combination of STDP and anti-STDP and proposed a remote supervised method (ReSuMe) algorithm that can learn spike train patterns for single layer SNNs. Using backpropagation of the spike train error, Sporea and Grüning [31] proposed the multi-ReSuMe algorithm to multilayer feedforward SNNs. Using the synaptic plasticity algorithms to train SNNs, the adjustment of synaptic weight only depends on the input and output spike trains and STDP mechanism, which is independent of neuron model and synaptic type. Therefore, these algorithms can be applied to various neuron models.

### 2.3. Supervised Learning Algorithms Based on Spike Train Convolution

Because the spike train is a discrete event set composed of the spikes of neurons, in order to facilitate analysis and calculation, a specific kernel function is selected, and the spike train is uniquely transformed into a continuous function by convolution method [32]. Through the convolution calculation of spike train based on kernel function, the spike train can be interpreted as specific neurophysiological signals, such as postsynaptic potential of neurons or density function of spike emissions [33]. Therefore, using the convolution representation of spike trains to construct the supervised learning algorithms will become an important direction for multilayer feedforward SNNs.

Carnell and Richardson [34] introduced a simple supervised learning algorithm of SNNs. According to the linear weighted representation of spike trains, the projection formula defined by Gram–Schmidt process is used to calculate the changes of synaptic weights. However, the algorithm has no error backpropagation mechanism and is only suitable for single-layer SNNs. Other spike train convolution algorithms for spiking neurons include spike pattern association neuron (SPAN) [35], precise-spike-driven (PSD) [36], and spike train kernel learning rule (STKLR) [37, 38]. Researchers have extended the SPAN and PSD learning algorithms for multilayer SNNs [39, 40]. Using the inner product representation of spike trains, the error function of spike trains and the relationship between input and output spike trains can be defined. Lin et al. [41] presented a new supervised learning algorithm for multilayer feedforward SNNs; its learning rules of synaptic weights in output and hidden layers are expressed as the spike train inner products, named multi-STIP.

Table 1 lists several typical supervised learning algorithms of multilayer feedforward SNNs. We compare these algorithms from the following three aspects: (1) the learning rules used for weight adjustment; (2) processing capability of information encoding, including spike train and single spike; and (3) applicability of spiking neuron models. The gradient descent algorithms are restricted to the spiking neuron models with analytical expressions, such as the SRM. However, some supervised learning algorithms are independent of the spiking neuron model used.

## 3. Neuron Model and Network Architecture

### 3.1. Long-Term Memory Spike Response Model

In the gradient descent learning algorithms for SNNs, the computation of partial derivatives is required, so the internal state of spiking neurons needs to be analyzed. SRM is widely used in the simulation of SNNs, especially in supervised learning because its internal state can be expressed analytically. In this paper, we consider the long-term memory SRM [10]. Assuming that the postsynaptic neuron *o* has *N*_*I*_ input presynaptic neurons, there are *N*_*i*_ spikes transmitted by the *i*th presynaptic neuron, and *t*_*i*_^*f*^ is the firing time of the *f*th spike (*f* ∈ [1, *F*_*i*_]). The membrane potential *u*_*o*_ can be described as follows:

(1) $$\begin{array}{c} u_{o}\left(t\right)=\sum_{i=1}^{N_{I}}\sum_{f=1}^{F_{i}}w_{oi}\varepsilon \left(t-t_{i}^{f}\right)+\sum_{r=1}^{F_{o}}\rho \left(t-t_{o}^{r}\right), \end{array}$$

where *w*_*oi*_ is the weight from the *i*th presynaptic neuron to the *o*th postsynaptic neuron, *t*_*o*_^*r*^ is the *r*th spike fired by the neuron *o*, and *F*_*o*_ is total number of spikes before the current time *t*.

The spike response function *ε* shows the influence of the presynaptic spike on the membrane potential of the postsynaptic neuron *o* and can be expressed as

(2) $$\begin{array}{c} \varepsilon \left(t-t_{i}^{f}\right)=\left\{\begin{array}{cc} \frac{t-t_{i}^{f}}{\tau }\exp\left(1-\frac{t-t_{i}^{f}}{\tau }\right), & t-t_{i}^{f}>0,\\ 0, & t-t_{i}^{f}\leq 0. \end{array}\right. \end{array}$$

After a neuron fired a spike, the membrane potential decreases rapidly to the resting potential. It is hard to fire a second spike within the refractory period. The refractoriness function *ρ* describes the effect of the current postsynaptic spike:

(3) $$\begin{array}{c} \rho \left(t-t_{o}^{r}\right)=\left\{\begin{array}{cc} -\theta \;\exp\left(-\frac{t-t_{o}^{r}}{\tau_{R}}\right), & t-t_{o}^{r}>0,\\ 0, & t-t_{o}^{r}\leq 0, \end{array}\right. \end{array}$$

where *τ* and *τ*_*R*_ are the time constants and *θ* is the threshold of membrane potential.

For a cumulative SRM neuron, when it fires multiple spikes during the given time interval, the effects of refractoriness can add up, which is a significant feature of long-term memory SRM. In formula (1), the combined effect of several previous spikes (*F*_*o*_ > 1) can produce spike frequency adaptation and intrinsic bursting [15, 16]. Therefore, long-term memory SRM neuron is more complex and biologically plausible than the SRM_0_ neuron model, in which refractoriness is modelled by only the most recent spike.

### 3.2. Multilayer Feedforward SNN Architecture

Multilayer feedforward SNN is a widely used topology architecture, where each neuron is only connected to the neurons in the previous layer. Spike trains are transmitted from the previous layer to the next layer through synapse connections. The input data of the specific problem are encoded into spike trains as the input information in a feedforward SNN. The neuronal activities of hidden layer neurons are triggered by the input spike trains. There may be one or more hidden layers in the feedforward SNN. The output layer represents the output of the network. In this paper, we consider a fully connected three-layer feedforward SNN, where any two neurons in adjacent layers are connected through a modifiable synaptic weight, as shown in Figure 1.

## 4. Supervised Learning Rules Based on Gradient Descent

### 4.1. Spike Train Error Function

In this paper, we use the spike times directly to construct the error function for SNNs. For the output neuron *o*, the actual output spike train is denoted as *s*_*o*_^*a*^={*t*_*o*_^1^, *t*_*o*_^2^,…, *t*_*o*_^*F*_*o*_^}, the desired output spike train is denoted as $s_{o}^{d}=\left\{{\hat{t}}_{o}^{1},{\hat{t}}_{o}^{2},\ldots ,{\hat{t}}_{o}^{F_{d}}\right\}$, and *F*_*o*_ and *F*_*d*_ are numbers of spikes in *s*_*o*_^*a*^ and *s*_*o*_^*d*^, respectively. The network error function can be defined as

(4) $$\begin{array}{c} E=\frac{1}{2}\sum_{o=1}^{N_{O}}\sum_{f=1}^{F}{\left(t_{o}^{f}-{\hat{t}}_{o}^{f}\right)}^{2}, \end{array}$$

where *N*_*O*_ is the neuron number of output layer and *F*=max{*F*_*o*_, *F*_*d*_} is the maximum of *F*_*o*_ and *F*_*d*_.

The spike number of spike train *s*_*o*_^*a*^ in different learning epochs may be different from the spike number in its desired spike train *s*_*o*_^*d*^. That is to say, *F*_*o*_ and *F*_*d*_ are not necessarily equal. We solve this problem according to the following strategies: (1) If *F*_*o*_ = *F*_*d*_, that is, *F* = *F*_*o*_ = *F*_*d*_, there is a one-to-one correspondence between *t*_*o*_^*a*^ and ${\hat{t}}_{o}^{d}$ in formula (4). (2) If *F*_*o*_ < *F*_*d*_, that is *F* = *F*_*d*_, the last spike *t*_*o*_^*F*_*o*_^ in *s*_*o*_^*a*^ is used to compute the error *E* with spikes ${\hat{t}}_{o}^{F_{o}},\ldots ,{\hat{t}}_{o}^{F_{d}}$ in *s*_*o*_^*d*^ that cannot be matched. (3) If *F*_*o*_ > *F*_*d*_, that is, *F* = *F*_*o*_, the last spike ${\hat{t}}_{o}^{F_{d}}$ in *s*_*o*_^*d*^ is used to compute the error *E* with spikes *t*_*o*_^*F*_*d*_^,…, *t*_*o*_^*F*_*o*_^ in *s*_*o*_^*a*^ that cannot be matched.

### 4.2. Synaptic Weight Learning Rules

This form of error function is helpful to deduce the synaptic weight updating rules by gradient descent method. The network error function is used to perform gradient calculation on the synaptic weights. According to the delta updating rule, the change of synaptic weight ∆*w* between the presynaptic and postsynaptic neurons is expressed as

(5) $$\begin{array}{c} \Delta w=-\eta \nabla E=\frac{\partial E}{\partial w}, \end{array}$$

where *η* is the learning rate. For the multilayer feedforward SNNs, the corresponding synaptic weight updating rules are different with the synapses in different layers.

(1) For the synaptic weight *w*_*oh*_ between the output neuron *o* and the hidden neuron *h*, using the chain rule, the gradient ∇*E*_*oh*_ can be calculated as follows:
  (6) $$\begin{array}{c} \nabla E_{oh}=\frac{\partial E}{\partial w_{oh}}=\sum_{f=1}^{F}\frac{\partial E}{\partial t_{o}^{f}}\frac{\partial t_{o}^{f}}{\partial w_{oh}}. \end{array}$$
According to the error function defined in formula (4), the partial derivative term ∂*E*/∂*t*_*o*_^*a*^ in formula (6) is determined by
  (7) $$\begin{array}{c} \frac{\partial E}{\partial t_{o}^{f}}=\frac{\partial \left[\left(1/2\right)\sum_{o=1}^{N_{O}}\sum_{f=1}^{F}{\left(t_{o}^{f}-{\hat{t}}_{o}^{f}\right)}^{2}\right]}{\partial t_{o}^{f}}=t_{o}^{f}-{\hat{t}}_{o}^{f} \end{array}$$
Using the chain rule again, the partial derivative term ∂*t*_*o*_^*f*^/∂*w*_*oh*_ in formula (6) is calculated as follows:
  (8) $$\begin{array}{c} \frac{\partial t_{o}^{f}}{\partial w_{oh}}=\frac{\partial t_{o}^{f}}{\partial u_{o}\left(t_{o}^{f}\right)}\frac{\partial u_{o}\left(t_{o}^{f}\right)}{\partial w_{oh}}. \end{array}$$
Based on [42], the partial derivative term ∂*t*_*o*_^*f*^/∂*u*_*o*_(*t*_*o*_^*f*^) in formula (8) is rewritten as
  (9) $$\begin{array}{c} \frac{\partial t_{o}^{f}}{\partial u_{o}\left(t_{o}^{f}\right)}=\frac{-1}{\partial u_{o}\left(t_{o}^{f}\right)/\partial t_{o}^{f}}. \end{array}$$
According to the long-term memory SRM expressed in formula (1), we can obtain the partial derivative term ∂*u*_*o*_(*t*_*o*_^*f*^)/∂*t*_*o*_^*f*^ as follows:
  (10) $$\begin{array}{c} \frac{\partial u_{o}\left(t_{o}^{f}\right)}{\partial t_{o}^{f}}=\sum_{h=1}^{N_{H}}\sum_{g=1}^{F_{h}}w_{oh}\varepsilon \left(t_{o}^{f}-t_{h}^{g}\right)\left(\frac{1}{t_{o}^{f}-t_{h}^{g}}-\frac{1}{\tau }\right)-\frac{1}{\tau_{R}}\sum_{t_{o}^{r}\in s_{o}^{a},t_{o}^{r}<t_{o}^{f}}\rho \left(t_{o}^{f}-t_{o}^{r}\right), \end{array}$$
where NH is the neuron number of hidden layer, *t*_*h*_^*g*^ is the *g*th spike fired by the hidden neuron *h*, and *t*_*o*_^*r*^ represents the recent spike in the spike train *s*_*o*_^*a*^ that is before *t*_*o*_^*f*^. Using formulas (9) and (10), the partial derivative term ∂*t*_*o*_^*f*^/∂*u*_*o*_(*t*_*o*_^*f*^) in formula (8) can be calculated as follows:
  (11) $$\begin{array}{c} \frac{\partial t_{o}^{f}}{\partial u_{o}\left(t_{o}^{f}\right)}=\frac{-1}{\sum_{h=1}^{N_{H}}\sum_{g=1}^{F_{h}}w_{oh}\varepsilon \left(t_{o}^{f}-t_{h}^{g}\right)\left(\left(1/\left(t_{o}^{f}-t_{h}^{g}\right)\right)-\left(1/\tau \right)\right)-\left(1/\tau_{R}\right)\sum_{t_{o}^{r}\in s_{o}^{a},t_{o}^{r}<t_{o}^{f}}\rho \left(t_{o}^{f}-t_{o}^{r}\right)}. \end{array}$$
According to the long-term memory SRM with cumulative refractoriness, the partial derivative term ∂*u*_*o*_(*t*_*o*_^*f*^)/∂*w*_*oh*_ in formula (8) can be calculated as follows:
  (12) $$\begin{array}{c} \frac{\partial u_{o}\left(t_{o}^{f}\right)}{\partial w_{oh}}=\sum_{g=1}^{F_{h}}\varepsilon \left(t_{o}^{f}-t_{h}^{g}\right)+\sum_{t_{o}^{r}\in s_{o}^{a},t_{o}^{r}<t_{o}^{f}}\frac{\partial \rho \left(t_{o}^{f}-t_{o}^{r}\right)}{\partial w_{oh}}. \end{array}$$
The recent output spike *t*_*o*_^*r*^ before *t*_*o*_^*f*^ in the refractoriness function is directly related to the membrane potential of the neuron, so it depends on the synaptic weight *w*_*oh*_. The partial derivative term ∂*ρ*(*t*_*o*_^*f*^ − *t*_*o*_^*r*^)/∂*w*_*oh*_ in formula (12) is calculated as follows:
  (13) $$\begin{array}{c} \frac{\partial \rho \left(t_{o}^{f}-t_{o}^{r}\right)}{\partial w_{oh}}=\frac{\partial \rho \left(t_{o}^{f}-t_{o}^{r}\right)}{\partial t_{o}^{r}}\frac{\partial t_{o}^{r}}{\partial w_{oh}}=\frac{1}{\tau_{R}}\rho \left(t_{o}^{f}-t_{o}^{r}\right)\frac{\partial t_{o}^{r}}{\partial w_{oh}}. \end{array}$$
The partial derivative term ∂*t*_*o*_^*r*^/∂*w*_*oh*_ can be calculated recursively using the following equations [14]:
  (14) $$\begin{array}{c} \frac{\partial t_{o}^{r}}{\partial w_{oh}}=\frac{\partial t_{o}^{r}}{\partial u_{o}\left(t_{o}^{r}\right)}\left[\frac{\partial u_{o}\left(t_{o}^{r}\right)}{\partial w_{oh}}+\frac{\partial u_{o}\left(t_{o}^{r}\right)}{\partial t_{o}^{r-1}}\frac{\partial t_{o}^{r-1}}{\partial w_{oh}}\right], \end{array}$$
  (15) $$\begin{array}{c} \frac{\partial t_{o}^{r-1}}{\partial w_{oh}}=\frac{\partial t_{o}^{r-1}}{\partial u_{o}\left(t_{o}^{r-1}\right)}\left[\frac{\partial u_{o}\left(t_{o}^{r-1}\right)}{\partial w_{oh}}+\frac{\partial u_{o}\left(t_{o}^{r-1}\right)}{\partial t_{o}^{r-2}}\frac{\partial t_{o}^{r-2}}{\partial w_{oh}}\right], \end{array}$$
  (16) $$\begin{array}{c} \frac{\partial t_{o}^{1}}{\partial w_{oh}}=\frac{\partial t_{o}^{1}}{\partial u_{o}\left(t_{o}^{1}\right)}\frac{\partial u_{o}\left(t_{o}^{1}\right)}{\partial w_{oh}}. \end{array}$$
The first and second partial derivative terms on the right-hand side of formula (16) have been calculated by formulas (11) and (12), respectively.
By substituting formulas (11) and (12) into formula (8), the partial derivative term ∂*t*_*o*_^*f*^/∂*w*_*oh*_ is calculated as follows:
  (17) $$\begin{array}{c} \frac{\partial t_{o}^{f}}{\partial w_{oh}}=\frac{-\sum_{g=1}^{F_{h}}\varepsilon \left(t_{o}^{f}-t_{h}^{g}\right)-\left(1/\tau_{R}\right)\sum_{t_{o}^{r}\in s_{o}^{a},t_{o}^{r}<t_{o}^{f}}\rho \left(t_{o}^{f}-t_{o}^{r}\right)\left(\partial t_{o}^{r}/\partial w_{oh}\right)}{\sum_{h=1}^{N_{H}}\sum_{g=1}^{F_{h}}w_{oh}\varepsilon \left(t_{o}^{f}-t_{h}^{g}\right)\left(\left(1/\left(t_{o}^{f}-t_{h}^{g}\right)\right)-\left(1/\tau \right)\right)-\left(1/\tau_{R}\right)\sum_{t_{o}^{r}\in s_{o}^{a},t_{o}^{r}<t_{o}^{f}}\rho \left(t_{o}^{f}-t_{o}^{r}\right)}. \end{array}$$
Thus, we can obtain the error gradient with respect to synaptic weight:
  (18) $$\begin{array}{c} \nabla E_{oh}=\sum_{f=1}^{F}\frac{-\left(t_{o}^{f}-{\hat{t}}_{o}^{f}\right)\left[\sum_{g=1}^{F_{h}}\varepsilon \left(t_{o}^{f}-t_{h}^{g}\right)+\left(1/\tau_{R}\right)\sum_{t_{o}^{r}\in s_{o}^{a},t_{o}^{r}<t_{o}^{f}}\rho \left(t_{o}^{f}-t_{o}^{r}\right)\left(\partial t_{o}^{r}/\partial w_{oh}\right)\right]}{\sum_{h=1}^{N_{H}}\sum_{g=1}^{F_{h}}w_{oh}\varepsilon \left(t_{o}^{f}-t_{h}^{g}\right)\left(\left(1/\left(t_{o}^{f}-t_{h}^{g}\right)\right)-\left(1/\tau \right)\right)-\left(1/\tau_{R}\right)\sum_{t_{o}^{r}\in s_{o}^{a},t_{o}^{r}<t_{o}^{f}}\rho \left(t_{o}^{f}-t_{o}^{r}\right)}. \end{array}$$
According to the above derivation process, the learning rule of synaptic weights between the output and hidden layers can be obtained using formulas (5) and (18). The partial derivative term ∂*t*_*o*_^*r*^/∂*w*_*oh*_ in formula (18) can be calculated recursively using formulas (14)–(16).
(2) For the synapse between the hidden neuron *h* and the input neuron *i*, using the chain rule, the gradient ∇*E*_*hi*_ with respect to synaptic weight *w*_*hi*_ is expressed as
  (19) $$\begin{array}{c} \nabla E_{hi}=\frac{\partial E}{\partial w_{hi}}=\sum_{g=1}^{F_{h}}\frac{\partial E}{\partial t_{h}^{g}}\frac{\partial t_{h}^{g}}{\partial w_{hi}}. \end{array}$$
Using the error function and chain rule, the partial derivative term ∂*E*/∂*t*_*h*_^*g*^ can be calculated as follows:
  (20) $$\begin{array}{c} \frac{\partial E}{\partial t_{h}^{g}}=\sum_{o=1}^{N_{O}}\sum_{f=1}^{F}\frac{\partial E}{\partial t_{o}^{f}}\frac{\partial t_{o}^{f}}{\partial u_{o}\left(t_{o}^{f}\right)}\frac{\partial u_{o}\left(t_{o}^{f}\right)}{\partial t_{h}^{g}}. \end{array}$$
The first and second partial derivative terms on the right-hand side of formula (20) have been calculated by formulas (7) and (11), respectively. According to the long-term memory SRM, the partial derivative term ∂*u*_*o*_(*t*_*o*_^*f*^)/∂*t*_*h*_^*g*^ can be calculated as follows:
  (21) $$\begin{array}{c} \frac{\partial u_{o}\left(t_{o}^{f}\right)}{\partial t_{h}^{g}}=-w_{oh}\varepsilon \left(t_{o}^{f}-t_{h}^{g}\right)\left(\frac{1}{t_{o}^{f}-t_{h}^{g}}-\frac{1}{\tau }\right)+\sum_{t_{o}^{r}\in s_{o}^{a},t_{o}^{r}<t_{o}^{f}}\frac{\partial \rho \left(t_{o}^{f}-t_{o}^{r}\right)}{\partial t_{h}^{g}}. \end{array}$$
The partial derivative term ∂*ρ*(*t*_*o*_^*a*^ − *t*_*o*_^*r*^)/∂*t*_*h*_^*g*^ in formula (21) can expressed as
  (22) $$\begin{array}{c} \frac{\partial \rho \left(t_{o}^{f}-t_{o}^{r}\right)}{\partial t_{h}^{g}}=\frac{\partial \rho \left(t_{o}^{f}-t_{o}^{r}\right)}{\partial t_{o}^{r}}\frac{\partial t_{o}^{r}}{\partial t_{h}^{g}}=\frac{1}{\tau_{R}}\rho \left(t_{o}^{f}-t_{o}^{r}\right)\frac{\partial t_{o}^{r}}{\partial t_{h}^{g}}. \end{array}$$
Thus, we can obtain ∂*E*/∂*t*_*h*_^*g*^ as follows:
  (23) $$\begin{array}{c} \frac{\partial E}{\partial t_{h}^{g}}=\sum_{o=1}^{N_{O}}\sum_{f=1}^{F}\frac{\left(t_{o}^{f}-{\hat{t}}_{o}^{f}\right)\left[w_{oh}\varepsilon \left(t_{o}^{f}-t_{h}^{g}\right)\left(\left(1/t_{o}^{f}-t_{h}^{g}\right)-\left(1/\tau \right)\right)-\left(1/\tau_{R}\right)\sum_{t_{o}^{r}\in s_{o}^{a},t_{o}^{r}<t_{o}^{f}}\rho \left(t_{o}^{f}-t_{o}^{r}\right)\left(\partial t_{o}^{r}/\partial t_{h}^{g}\right)\right]}{\sum_{h=1}^{N_{H}}\sum_{g=1}^{F_{h}}w_{oh}\varepsilon \left(t_{o}^{f}-t_{h}^{g}\right)\left(\left(1/\left(t_{o}^{f}-t_{h}^{g}\right)\right)-\left(1/\tau \right)\right)-\left(1/\tau_{R}\right)\sum_{t_{o}^{r}\in s_{o}^{a},t_{o}^{r}<t_{o}^{f}}\rho \left(t_{o}^{f}-t_{o}^{r}\right)}. \end{array}$$
The output spike *t*_*o*_^*r*^ is dependent on the previous output spikes because of the existence of the cumulative refractoriness function. Using the recursive equations, the partial derivative term ∂*t*_*o*_^*r*^/∂*t*_*h*_^*g*^ in formula (23) can be calculated as follows:
  (24) $$\begin{array}{c} \frac{\partial t_{o}^{r}}{\partial t_{h}^{g}}=\frac{\partial t_{o}^{r}}{\partial u_{o}\left(t_{o}^{r}\right)}\left[\frac{\partial u_{o}\left(t_{o}^{r}\right)}{\partial t_{h}^{g}}+\frac{\partial u_{o}\left(t_{o}^{r}\right)}{\partial t_{o}^{r-1}}\frac{\partial t_{o}^{r-1}}{\partial t_{h}^{g}}\right], \end{array}$$
  (25) $$\begin{array}{c} \frac{\partial t_{o}^{r-1}}{\partial t_{h}^{g}}=\frac{\partial t_{o}^{r-1}}{\partial u_{o}\left(t_{o}^{r-1}\right)}\left[\frac{\partial u_{o}\left(t_{o}^{r-1}\right)}{\partial t_{h}^{g}}+\frac{\partial u_{o}\left(t_{o}^{r-1}\right)}{\partial t_{o}^{r-2}}\frac{\partial t_{o}^{r-2}}{\partial t_{h}^{g}}\right], \end{array}$$
  (26) $$\begin{array}{c} \frac{\partial t_{o}^{1}}{\partial t_{h}^{g}}=\frac{\partial t_{o}^{1}}{\partial u_{o}\left(t_{o}^{1}\right)}\frac{\partial u_{o}\left(t_{o}^{1}\right)}{\partial t_{h}^{g}}. \end{array}$$
The first and second partial derivative terms on the right-hand side of formula (26) have been calculated by formulas (11) and (21), respectively.
The partial derivative term ∂*t*_*h*_^*g*^/∂*w*_*hi*_ in formula (19) can be expressed using the chain rule:
  (27) $$\begin{array}{c} \frac{\partial t_{h}^{g}}{\partial w_{hi}}=\frac{\partial t_{h}^{g}}{\partial u_{h}\left(t_{h}^{g}\right)}\frac{\partial u_{h}\left(t_{h}^{g}\right)}{\partial w_{hi}}. \end{array}$$
Similar to formula (9), the partial derivative term ∂*t*_*h*_^*g*^/∂*u*_*h*_(*t*_*h*_^*g*^) can be calculated as follows:
  (28) $$\begin{array}{c} \frac{\partial t_{h}^{g}}{\partial u_{h}\left(t_{h}^{g}\right)}=\frac{-1}{\partial u_{h}\left(t_{h}^{g}\right)/\partial t_{h}^{g}}=\frac{-1}{\sum_{i=1}^{N_{I}}\sum_{k=1}^{F_{i}}w_{hi}\varepsilon \left(t_{h}^{g}-t_{i}^{k}\right)\left(\left(1/\left(t_{h}^{g}-t_{i}^{k}\right)\right)-\left(1/\tau \right)\right)-\left(1/\tau_{R}\right)\sum_{t_{h}^{r}\in s_{h},t_{h}^{r}<t_{h}^{g}}\rho \left(t_{h}^{g}-t_{h}^{r}\right)}, \end{array}$$
where *N*_*I*_ is the number of input neurons, *t*_*i*_^*k*^ is the *k*th spike fired by the neuron *i*, and *t*_*h*_^*r*^ represents the recent spike in the spike train *s*_*h*_ that is before *t*_*h*_^*g*^. The partial derivative term ∂*u*_*h*_(*t*_*h*_^*g*^)/∂*w*_*hi*_ in formula (27) can be calculated as follows:
  (29) $$\begin{array}{c} \frac{\partial u_{h}\left(t_{h}^{g}\right)}{\partial w_{hi}}=\sum_{k=1}^{F_{i}}\varepsilon \left(t_{h}^{g}-t_{i}^{k}\right)+\frac{1}{\tau_{R}}\sum_{t_{h}^{r}\in s_{h},t_{h}^{r}<t_{h}^{g}}\rho \left(t_{h}^{g}-t_{h}^{r}\right)\frac{\partial t_{h}^{r}}{\partial w_{hi}}. \end{array}$$
The partial derivative term ∂*t*_*h*_^*r*^/∂*w*_*hi*_ can be also calculated as formulas (14)–(16). By substituting formulas (28) and (29) into formula (27), we can obtain
  (30) $$\begin{array}{c} \frac{\partial t_{h}^{g}}{\partial w_{hi}}=\frac{-\sum_{k=1}^{F_{i}}\varepsilon \left(t_{h}^{g}-t_{i}^{k}\right)-\left(1/\tau_{R}\right)\sum_{t_{h}^{r}\in s_{h},t_{h}^{r}<t_{h}^{g}}\rho \left(t_{h}^{g}-t_{h}^{r}\right)\left(\partial t_{h}^{r}/\partial w_{hi}\right)}{\sum_{i=1}^{N_{I}}\sum_{k=1}^{F_{i}}w_{hi}\varepsilon \left(t_{h}^{g}-t_{i}^{k}\right)\left(\left(1/\left(t_{h}^{g}-t_{i}^{k}\right)\right)-\left(1/\tau \right)\right)-\left(1/\tau_{R}\right)\sum_{t_{h}^{r}\in s_{h},t_{h}^{r}<t_{h}^{g}}\rho \left(t_{h}^{g}-t_{h}^{r}\right)}. \end{array}$$

According to the above derivation process, the gradient ∇*E*_*hi*_ can be obtained by substituting formulas (23) and (30) into formula (19). The update values of synaptic weights between the hidden and input layers can be calculated by formula (5) and the gradient ∇*E*_*hi*_. The partial derivative term ∂*t*_*o*_^*r*^/∂*t*_*h*_^*g*^ in formula (23) can be calculated recursively using formulas (24)–(26). The partial derivative term ∂*t*_*h*_^*r*^/∂*w*_*hi*_ in formula (30) can be calculated by the similar recursive formulas (14)–(16).

### 4.3. Computational Complexity Analysis of the Algorithm

The computational complexity of the proposed supervised learning algorithm depends on the SNN scale and spike firing rate of neurons. For simplicity of analysis, we choose a three-layer feedforward SNN. We assume that the number of neurons in the different layers is *N*_*I*_, *N*_*H*_, and *N*_*O*_, respectively, and the average spike number of neurons is ${\bar{F}}_{N}$ in the given simulation duration. According to the above deduced learning rules of SNNs with long-term memory SRM, the computing time of synaptic weight adjustment mainly determined by the number of calls of the spike response function *ε* and the refractoriness function *ρ*. Both *ε* (formula (2)) and *ρ* (formula (3)) functions are exponential functions, which are regarded as basic operations. Therefore, the number of exponential function calls is used to measure time complexity of learning algorithm. Assuming that *C*_*F*_ represents the computation time of each basic operation, the computational complexity of different layer learning rules is analyzed as follows:

(1) As shown in formula (6), for the synaptic weight *w*_*oh*_ between the output neuron *o* and the hidden neuron *h*, its update value is accumulated by the effects of output spikes. By way of recurrence, the partial derivative term ∂*t*_*o*_^*r*^/∂*w*_*oh*_ is computed using the mode in which previous values are stored. The calculation time cost for each spike *t*_*o*_^*f*^ of the output neuron is expressed as
  (31) $$\begin{array}{c} \left[N_{H}{\bar{F}}_{H}\left(t_{o}^{f}\right)+2F_{o}\left(t_{o}^{f}\right)+F_{h}\left(t_{o}^{f}\right)\right]C_{F}, \end{array}$$
where ${\bar{F}}_{H}\left(t_{o}^{f}\right)$ is the average spike number of the hidden neurons that fire spikes before *t*_*o*_^*f*^ and *F*_*o*_(*t*_*o*_^*f*^) and *F*_*h*_(*t*_*o*_^*f*^) are the number of spikes fired before *t*_*o*_^*f*^ for the output neuron *o* and the hidden neuron *h*, respectively. The weight updating calculation of all output spikes is accumulated; the asymptotic time complexity is $O\left(N_{H}{\bar{F}}_{N}{}^{2}C_{F}\right)$ for the update of synaptic weight *w*_*oh*_. Therefore, the total time complexity of all synaptic weight adjustments between the output and hidden layers is $O\left(N_{O}N_{H}^{2}{\bar{F}}_{N}{}^{2}C_{F}\right)$.
(2) As shown in formula (19), for the synaptic weight *w*_*hi*_ between the hidden neuron *h* and the input neuron *i*, its update value is accumulated by the effects of hidden spikes. The partial derivative terms ∂*t*_*o*_^*r*^/∂*t*_*h*_^*g*^ and ∂*t*_*h*_^*r*^/∂*w*_*hi*_ are also computed using the recursive and storage mode. For each spike *t*_*h*_^*g*^ of the output neuron, the calculation time cost of the partial derivative term ∂*E*/∂*t*_*h*_^*g*^ is expressed as
  (32) $$\begin{array}{c} \sum_{o=1}^{N_{O}}\sum_{f=1}^{F}\left[N_{H}{\bar{F}}_{H}\left(t_{o}^{f}\right)+2F_{o}\left(t_{o}^{f}\right)+1\right]C_{F}. \end{array}$$

The calculation time cost of the partial derivative term ∂*t*_*h*_^*g*^/∂*w*_*hi*_ is expressed as

(33) $$\begin{array}{c} \left[N_{I}{\bar{F}}_{I}\left(t_{h}^{g}\right)+2F_{h}\left(t_{h}^{g}\right)+F_{i}\left(t_{h}^{g}\right)\right]C_{F}, \end{array}$$

where ${\bar{F}}_{I}\left(t_{h}^{g}\right)$ is the average spike number of the input neurons that fire spikes before *t*_*h*_^*g*^ and *F*_*h*_(*t*_*h*_^*g*^) and *F*_*i*_(*t*_*h*_^*g*^) are the number of spikes fired before *t*_*h*_^*g*^ for the hidden neuron *h* and the input neuron *i*, respectively. Accumulating the effects of all spikes of hidden neuron *h*, the asymptotic time complexity is $O\left(N_{O}N_{H}{\bar{F}}_{N}{}^{3}C_{F}+N_{I}{\bar{F}}_{N}{}^{2}C_{F}\right)$ for the update of synaptic weight *w*_*hi*_. The number of weights between the hidden and input layers is *N*_*H*_*N*_*I*_ in the fully connected networks, so the total asymptotic time complexity of all synaptic weight adjustments is $O\left(N_{O}N_{H}^{2}N_{I}{\bar{F}}_{N}{}^{3}C_{F}+N_{H}N_{I}^{2}{\bar{F}}_{N}{}^{2}C_{F}\right)$.

## 5. Result Analysis and Discussion

### 5.1. Parameter Settings

In the simulation, the clock-driven simulation strategy is employed to perform the spike train learning, where the time step is *dt* = 0.1 ms. The long-term memory SRM described in Section 3.1 is used in all experiments. The parameter values of the long-term memory SRM are set as follows: the spike response time constant *τ* = 3 ms, the refractoriness time constant *τR* = 35 ms, the absolute refractory period *tref* = 1 ms, and the threshold of neuronal spike firing *θ* = 1. The three-layer feedforward SNN is fully connected; the number of neurons in the input layer, the hidden layer, and the output layer is *NI* = 50, *NH* = 130, and *NO* = 1, respectively. The length of SNN simulation is Γ = 100 ms, the firing rate is 30 Hz for the input and desired output spike trains, and the input and desired output spike trains are generated by Poisson's process. The synaptic weight between two neurons is generated randomly in the interval [0, 0.2]. In the learning process of SNN, the learning rate of the proposed algorithm is set as *η* = 0.005. The upper limit of learning epoch is 300. Unless otherwise specified, each experiment is performed 50 trials, and the training results are averaged. The multi-ReSuMe algorithm [31] for multilayer feedforward SNN can achieve spike train learning. So, we compare our proposed algorithm with multi-ReSuMe in the learning tasks of spike trains using the long-term memory SRM. For the multi-ReSuMe algorithm, its learning rate is 0.5. The correlation-based metric *C* is often used for evaluating the similarity of spike trains [43]; it can also be used to evaluate the spike train learning capability of the supervised learning algorithms.

### 5.2. Spike Train Learning

Firstly, the process of learning sequences of spikes is analyzed using the proposed algorithm.  Figure 2 shows the spike train learning process of a SNN with 150 hidden neurons to match the desired output spike train. The evolution of actual output spike train in the training process is shown in Figure 2(a). With the change of learning epoch, the actual spike train fired by the output neuron gradually approaches the desired spike train.  Figure 2(b) shows the change trend of learning accuracy during the learning process. It indicates that learning accuracy C increased gradually during the learning process and reached 1.0 after 40 learning epochs. The changes of synaptic weights between the output and hidden neurons are also analyzed.  Figure 2(c) shows the weight values before training, and Figure 2(d) shows the weight values after training. This simulation indicates that our method can successfully train the feedforward SNN to learn spike trains.

Next, the effects of network scale parameters on learning performance are analyzed and compared with the multi-ReSuMe algorithm. The influence of the number of input neurons is shown in Figures 3(a) and 3(b); the input neuron number increases from 30 to 210 in steps of 20.  Figure 3(a) shows that the learning accuracy of two algorithms increases gradually along with the increasing of input neurons. However, the proposed method can achieve higher learning accuracy than multi-ReSuMe. When the number of input neurons is 150, the learning accuracy of our proposed algorithm is *C* = 0.9563, which is higher than *C* = 0.9447 for multi-ReSuMe.  Figure 3(b) represents the learning epochs when the training algorithm achieves the highest learning accuracy. It shows that the learning epochs of the proposed learning algorithm are less than those of multi-ReSuMe. For example, the learning epochs of our proposed algorithm and multi-ReSuMe are 194.28 and 258.74, respectively, for the 110 input neurons. Figures 3(c) and 3(d) show the learning results when the number of hidden neurons increases from 40 to 310 in steps of 30. The change trend of learning accuracy and epochs are similar to that of the increasing of input neurons. For example, when the number of hidden neurons is 130, the learning accuracy of our proposed algorithm is *C* = 0.9824 and the learning accuracy of multi-ReSuMe is *C* = 0.9582. When the training algorithms achieve the highest learning accuracy, the learning epochs of two algorithms are 248.49 and 264.28 for the 220 hidden neurons. Therefore, with the increase of SNN scale, two supervised learning algorithms have stronger spike train learning ability.

Finally, the effects of the spike train parameters on learning performance are analyzed and compared with the multi-ReSuMe algorithm. Figures 4(a) and 4(b) show that the learning results with the change of spike firing rate; it increases from 20 Hz to 110 Hz in steps of 10 Hz. As shown in Figure 4(a), the learning accuracy of the two algorithms decreases gradually with the increasing of the firing rate of spike trains. However, the proposed method can achieve higher learning accuracy than multi-ReSuMe. For example, when the spike train firing rate is 40 Hz, the learning accuracy of our method is 0.9824, and *C* = 0.9174 for the multi-ReSuMe algorithm.  Figure 4(b) represents the learning epochs when the training algorithm achieves the highest learning accuracy. It shows that the learning epochs of both our method and multi-ReSuMe increase firstly and then decrease with the increasing of the spike firing rate, and the proposed learning algorithm has less learning epochs. For example, the learning epochs of two algorithms are 182.46 and 218.49 when the firing rate spike trains is 50 Hz. When the length of spike trains increases from 50 ms to 500 ms in steps of 50 ms, the learning results are shown in Figures 4(c) and 4(d). The learning accuracy and epochs have a downward trend with the increase of the spike train length. For example, when the spike train length is 150 ms, the learning accuracy of our method and the multi-ReSuMe is *C* = 0.9675 and *C* = 0.9231, respectively. When the spike train length is 350 ms, the learning epochs of the two algorithms are 180.78 and 217.74, respectively. Therefore, when the spike train is more complex, the optimization of synaptic weights in the SNN is more difficult.

### 5.3. Nonlinear Pattern Classification

The proposed method is also used to solve actual nonlinear pattern classification problems in the multilayer feedforward SNNs. We select the 4 benchmark datasets: Fisher Iris, Pima Indians Diabetes (PIMA), Wisconsin Breast Cancer (WBC), and Liver Disorders; these classification problems are from the UCI machine learning library [44]. The samples are divided into training and testing sets.  Table 2 shows the details of benchmark datasets.

Each feature value of samples in the 4 datasets is normalized and converted into the frequency interval of [30, 50] Hz. Using a linear encoding method, each frequency value is then encoded as a spike train within [0, 50] ms. For the 4 datasets, the range of the initial synaptic weights before learning and the time constant *τ* of the postsynaptic potential of the long-term memory SRM are different. Also, the label information of each sample in the 4 datasets is encoded into desired spike trains with different frequencies using a linear encoding scheme.  Table 3 shows the parameter settings for different datasets. In this experiment, each result is averaged over 20 trials. We compare our proposed algorithm with the multi-STIP [41] and multi-ReSuMe [31] algorithms using the long-term memory SRM on classification performance. The learning rates of these 3 algorithms for the nonlinear pattern classification problems are shown in Table 4.

Figure 5 shows the classification process of the supervised learning algorithms of SNNs for the Iris dataset. The number of misclassified samples on the training set trained with our method is shown in Figure 5(a). We note that the misclassified number of Versicolor samples decreases rapidly, and the misclassified samples of Setosa and Virginica do not change too much during the training process. When the learning epoch exceeds 20, the misclassification of the three kinds of samples will be gradually stable.  Figure 5(b) shows the evolution of the classification accuracy of our method, multi-STIP, and multi-ReSuMe on the training set. It shows that our method is more stable and can achieve higher classification accuracy than the other two supervised learning algorithms on the training set. On average, using our method to train SNNs, Setosa samples are classified correctly; 0.4 Versicolor samples and 1.4 Virginica samples are misclassified. Finally, the classification accuracy of our method, multi-STIP, and multi-ReSuMe is 97.6%, 96.1%, and 87.4%, respectively.

Figure 6 shows the classification results of an experiment for the PIMA dataset. As shown in Figure 6(a), the number of misclassified samples are obtained by training a SNN with our method. From Figure 6(a), it can be seen that the misclassified number of normal samples increases firstly and then decreases gradually, and the misclassified samples of sick decrease rapidly and then increase gradually during the training process. However, the overall number of misclassified samples is decreased.  Figure 6(b) shows the classification accuracy of three supervised learning algorithms on the training set. It shows that our method can achieve higher classification accuracy than multi-STIP and multi-ReSuMe. The average results are obtained over 20 trials using our method; the number of misclassified samples of normal and sick is 67.2 and 49.9, respectively. The mean classification accuracy of our method, multi-STIP, and multi-ReSuMe on the training set is 69.5%, 67.7%, and 66.7%, respectively.

Figure 7 shows the classification process of our method, multi-STIP, and multi-ReSuMe for the WBC dataset. The number of misclassified samples trained with our method is shown in Figure 7(a). It indicates that the misclassified number of benign samples increases gradually, and the misclassified number of malignant samples decreases rapidly during the training process. The overall number of misclassified samples is decreased gradually. Eventually, on average, 3.3 samples of benign tumor and 12.8 samples of malignant tumor are misclassified. The classification accuracy of three learning algorithms on the training set is shown in Figure 8(b). The classification accuracy of multi-STIP is the highest, our method is second, and multi-ReSuMe is the lowest. Through the average of 20 experiments, the classification accuracy of three methods on the training set is 95.3%, 96.1%, and 93.7%, respectively.

Figure 8 shows the classification process of an experiment using our method, multi-STIP, and multi-ReSuMe for the Liver dataset. As shown in Figure 8(a), the misclassified number of sick samples increases gradually, and the misclassified number of normal samples decreases during the training process using our method. The misclassified number tends to stable after 30 learning epochs. Figure 8(b) shows the evolution of classification accuracy of three supervised learning algorithms on the training set. It indicates that our method can achieve the highest classification accuracy. Eventually, on average, 32.4 samples of normal and 21.7 samples of sick are misclassified, and the classification accuracy of three methods on the training set is 68.1%, 62.4%, and 61.7%, respectively.

In order to verify the pattern classification ability of the proposed algorithm, the classification accuracy is compared against several other supervised learning algorithms using multilayer feedforward SNNs.  Table 5 shows the comparison results of classification accuracy of different methods for the datasets of Iris, PIMA, WBC, and Liver. The gradient descent algorithm SpikeProp [11] with single spike is chosen; synaptic plasticity algorithms SWAT [29] and multi-ReSuMe [31] and spike train convolution algorithm multi-STIP [41] are also chosen for comparison. The classification accuracy of SpikeProp and SWAT on the Iris and WBC datasets refers to the results described in [29], while the classification accuracy of SpikeProp and SWAT on the PIMA and Liver datasets refers to the results described in [45]. The classification accuracy of multi-ReSuMe, multi-STIP, and our method for the datasets of Iris, PIMA, WBC, and Liver is obtained by multilayer feedforward SNNs with long-term memory SRM.

As shown in Table 5, for the Iris dataset, the classification accuracy of our method is the highest; the training and testing classification accuracy is 97.6% and 97.2%, respectively. For the PIMA dataset, the classification accuracy of our method on the training and testing sets is 69.5% and 71.8%; it is higher than multi-STIP and multi-ReSuMe, but lower than SpikeProp and SWAT. For the WBC dataset, the classification accuracy of the proposed algorithm is 95.3% on the training set and 94.9% on the testing set, our method can achieve higher classification accuracy than the multi-ReSuMe algorithm. For the Liver dataset, the classification accuracy of the proposed algorithm is higher than that of multi-ReSuMe and multi-STIP on the training set and higher than that of SWAT, multi-ReSuMe, and multi-STIP on the testing set. The classification accuracy of our method is 68.1% and 64.7% on the training and testing sets, respectively. In general, our proposed algorithm adopts the simpler SNN structure and spike train encoding method; it can solve the nonlinear pattern classification problems well and achieve rather good results for different datasets.

## 6. Conclusions

Gradient descent rule is a conventional mathematical basis for designing learning algorithms of neural networks. The SNNs represent information by discrete spike times, which results in the related variables of neurons to the error function that is not continuously differentiable. So, the traditional error backpropagation method is not suitable for training SNNs. This paper presents a supervised learning algorithm based on gradient descent rule for multilayer feedforward SNNs, which can realize spike train learning. The feedforward network consists of spiking neurons governed by biologically plausible long-term memory SRM, in which the effect of earlier spikes on the refractoriness is not neglected to express the bursting and adaptation characteristics. Using the recursive equations, the gradient descent rules of different layers are derived to update synaptic weights. The extended SpikeProp algorithm with the long-term memory SRM can learn spike train in the input and hidden layers, but still limits the output neuron to fire single spike [17]. However, the advantage of the proposed algorithm can learn spike trains in all layers.

The proposed algorithm is performed on some spike train learning tasks with various parameters. The results indicate that our method can obtain higher learning accuracy and less learning epochs in comparison with the multi-ReSuMe algorithm. Some important parameters of network simulation are analyzed; it is shown that the proposed algorithm is robust for a large parameter space. In addition, the proposed algorithm is used to solve the nonlinear pattern classification problems on UCI benchmark datasets of Iris, PIMA, WBC, and Liver. Experimental results show that our method can well solve the nonlinear pattern classification problems and achieve high classification accuracy for different datasets in comparison to other algorithms for multilayer feedforward SNNs. The proposed learning algorithm runs in an offline manner. It needs to study the online gradient descent learning algorithms for multilayer feedforward SNNs and use them to solve real-time pattern recognition problems in an online manner.

## Figures and Tables

**Figure 1:** Architecture of a multilayer feedforward SNN.

**Figure 2:** The learning process of spike train trained with our method. (a) The evolution of actual spike train of the output neuron in the training process. ▽ and • represent the desired and actual output spikes during the training process, and △ represents the initial output spikes before learning. (b) The change trend of learning accuracy. (c) The synaptic weight values before training. (d) The synaptic weight values after training.

**Figure 3:** The learning results of our method and multi-ReSuMe with the changes of network scale parameters. (a) The learning accuracy with different number of input neurons. (b) The learning epochs with different numbers of input neurons. (c) The learning accuracy with different numbers of hidden neurons. (d) The learning epochs with different numbers of hidden neurons.

**Figure 4:** The learning results of our method and multi-ReSuMe with the changes of spike train parameters. (a) The learning accuracy with different firing rates of spike trains. (b) The learning epochs with different firing rates of spike trains. (c) The learning accuracy with different lengths of spike trains. (d) The learning epochs with different lengths of spike trains.

**Figure 5:** Classification process of our method, multi-STIP, and multi-ReSuMe for the Iris dataset. (a) The number of misclassified samples trained with our method. (b) The evolution of the classification accuracy of three algorithms on the training set.

**Figure 6:** Classification process of our method, multi-STIP, and multi-ReSuMe for the PIMA dataset. (a) The number of misclassified samples trained with our method. (b) The evolution of the classification accuracy of three algorithms on the training set.

**Figure 7:** Classification process of our method, multi-STIP, and multi-ReSuMe for the WBC dataset. (a) The number of misclassified samples trained with our method. (b) The evolution of the classification accuracy of three algorithms on the training set.

**Figure 8:** Classification process of our method, multi-STIP, and multi-ReSuMe for the Liver dataset. (a) The number of misclassified samples trained with our method. (b) The evolution of the classification accuracy of three algorithms on the training set.

**Table 1:** Comparison of several typical supervised learning algorithms for multilayer feedforward SNNs.

Authors/Algorithm	Learning rule	Information encoding	Spiking neuron model
Bohte et al./SpikeProp [11]	Gradient descent rule	Single spike	The simplified SRM_0_
Xu et al./multi-SpikeProp [14]	Gradient descent rule	Spike train	The simplified SRM_0_
Booij and tat Nguyen/extended SpikeProp [17]	Gradient descent rule	Single spike	Long-term memory SRM
Zenke and Ganguli/SuperSpike [27]	Gradient descent rule	Spike train	Leaky integrate-and-fire model
Wade et al./SWAT [29]	STDP rule	Linear encoded spike train	Leaky integrate-and-fire model
Sporea and Grüning/multi-ReSuMe [31]	STDP rule	Spike train	Various spiking neuron models
Zhang et al./multi-SPAN [39]	Spike train convolution	Spike train	Various spiking neuron models
Lin et al./multi-STIP [41]	Spike train inner products	Spike train	Various spiking neuron models

**Table 2:** Description of datasets used for validation.

Dataset	Feature	Class	Number of samples in the training set	Number of samples in the testing set
Iris	4	3	75	75
PIMA	8	2	384	384
WBC	9	2	342	341
Liver	6	2	170	175

**Table 3:** Parameter settings for different datasets.

Dataset	Range of synaptic weights	Time constant *τ* (ms)	Firing rate of desired spike trains for different classes (Hz)	Upper limit of learning epochs
Iris	[0, 0.6]	7	30, 35, 40	150
PIMA	[0, 0.3]	9	30, 38	100
WBC	[0, 1.0]	9	32, 38	100
Liver	[0, 1.2]	3	30, 34	50

**Table 4:** Learning rates of our method, multi-STIP, and multi-ReSuMe for different datasets.

Dataset	Our method	Multi-STIP	Multi-ReSuMe
Iris	0.005	0.001	0.001
PIMA	0.001	0.0001	0.0001
WBC	0.0001	0.005	0.005
Liver	0.0001	0.0005	0.0005

**Table 5:** Comparison of classification accuracy of different methods for the 4 datasets.

Dataset	Algorithm	SNN architecture	Training accuracy	Testing accuracy
Iris	SpikeProp [29]	50–10–3	97.4% ± 0.1	96.1% ± 0.1
	SWAT [29]	16–208–3	95.5% ± 0.6	95.3% ± 3.6
	Multi-ReSuMe	4–80–1	87.4% ± 0.1	86.3% ± 0.8
	Multi-STIP	4–80–1	96.1% ± 1.1	94.2% ± 2.0
	Our method	4–80–1	97.6% ± 2.0	97.2% ± 2.0

PIMA	SpikeProp [45]	49–20–2	78.6% ± 2.5	76.2% ± 1.8
	SWAT [45]	48–624–2	77.0% ± 2.1	72.1% ± 1.8
	Multi-ReSuMe	8–100–1	66.7% ± 1.0	66.4% ± 0.9
	Multi-STIP	8–100–1	67.7% ± 2.0	69.5% ± 1.0
	Our method	8–100–1	69.5% ± 2.4	71.8% ± 1.4

WBC	SpikeProp [29]	64–15–2	97.6% ± 0.2	97.0% ± 0.6
	SWAT [29]	9–117–2	96.2% ± 0.4	96.7% ± 2.3
	Multi-ReSuMe	9–50–1	93.7% ± 1.0	94.4% ± 1.4
	Multi-STIP	9–50–1	96.1% ± 0.4	96.7% ± 0.7
	Our method	9–50–1	95.3% ± 0.6	94.9% ± 1.1

Liver	SpikeProp [45]	37–15–2	71.5% ± 5.2	65.1% ± 4.7
	SWAT [45]	36–468–2	74.8% ± 2.1	60.9% ± 3.2
	Multi-ReSuMe	6–50–1	61.8% ± 1.0	61.5% ± 1.4
	Multi-STIP	6–50–1	62.4% ± 2.0	60.8% ± 2.0
	Our method	6–50–1	68.1% ± 4.1	64.7% ± 2.7

## Data Availability

The supervised classification dataset benchmarks used to support the findings of this study have been taken from the UCI Machine Learning Repository of the University of California, Irvine (http://archive.ics.uci.edu/ml/index.php).
